The article "Arithmetic Optimization with RetinaNet Model for Motor Imagery Classification on Brain Computer Interface" was published in 2022. Journal: J Healthc Eng.

# Arithmetic Optimization with RetinaNet Model for Motor Imagery Classification on Brain Computer Interface

**DOI:** 10.1155/2022/3987494

**Published:** 2022-03-24

**Authors:** Areej A. Malibari, Fahd N. Al-Wesabi, Marwa Obayya, Mimouna Abdullah Alkhonaini, Manar Ahmed Hamza, Abdelwahed Motwakel, Ishfaq Yaseen, Abu Sarwar Zamani

**Affiliations:** ^1^Department of Industrial and Systems Engineering, College of Engineering,Princess Nourah Bint Abdulrahman University, P.O. Box 84428, Riyadh 11671, Saudi Arabia; ^2^Department of Computer Science, College of Science & Art at Mahayil, King Khalid University, Saudi Arabia; ^3^Department of Biomedical Engineering, College of Engineering, Princess Nourah Bint Abdulrahman University, P.O. Box 84428, Riyadh 11671, Saudi Arabia; ^4^Department of Computer Science, College of Computer and Information Sciences, Prince Sultan University, Saudi Arabia; ^5^Department of Computer and Self Development, Preparatory Year Deanship, Prince Sattam Bin Abdulaziz University, AlKharj, Saudi Arabia

## Abstract

Brain Computer Interface (BCI) technology commonly used to enable communication for the person with movement disability. It allows the person to communicate and control assistive robots by the use of electroencephalogram (EEG) or other brain signals. Though several approaches have been available in the literature for learning EEG signal feature, the deep learning (DL) models need to further explore for generating novel representation of EEG features and accomplish enhanced outcomes for MI classification. With this motivation, this study designs an arithmetic optimization with RetinaNet based deep learning model for MI classification (AORNDL-MIC) technique on BCIs. The proposed AORNDL-MIC technique initially exploits Multiscale Principal Component Analysis (MSPCA) approach for the EEG signal denoising and Continuous Wavelet Transform (CWT) is exploited for the transformation of 1D-EEG signal into 2D time-frequency amplitude representation, which enables to utilize the DL model via transfer learning approach. In addition, the DL based RetinaNet is applied for extracting of feature vectors from the EEG signal which are then classified with the help of ID3 classifier. In order to optimize the classification efficiency of the AORNDL-MIC technique, arithmetical optimization algorithm (AOA) is employed for hyperparameter tuning of the RetinaNet. The experimental analysis of the AORNDL-MIC algorithm on the benchmark data sets reported its promising performance over the recent state of art methodologies.

## 1. Introduction

Brain-computer interface (BCI) is a technology that permits us to communicate with the computer, whereby the device forecasts the abstract aspect of cognitive states with brain signals, namely, electroencephalography (EEG). Also, it is named as Brain-computer interface (BCI) that is commonly associated with AI-enabled approach which permits the user to harness brain, etc [1]. It is a noninvasive approach that gathers brain oscillatory activation patterns from the scalp. The human brain produces electrical signal that is identified by using EEG. Therefore, it is highly reliable and applicable method for receiving the control command for BCI [2]. Studies involving EEG signals when imagining limb or finger movement, widely called motor imagery (MI), to function artificial intelligence (AI) technique has been witnessed in this study [3]. An effective BCI scheme has two fundamental needs that consist of effective machine learning (ML) method for the classification of feature extraction and an efficient set of EEG feature must be capable of differentiating task induced brain activities. The study aims to identify the MI-task induced EEG patterns [4, 5].

Mostly, BCI system involves filtering or preprocessing to remove this undesirable component that is embedded with the EEG signals which leads to wrong conclusions and bias the analysis of the EEG [6]. Appropriate preprocessing within the BCI scheme results in cleaner EEG signal, thus enhancing the classification outcomes. The study focuses on the quantum mechanics inspired preprocessing phase within the BCI scheme, for extracting further data from the attained noisy EEG signal, and leads to increased classification performance although categorized by using multiple classification methods [7]. Especially, SVM is widely employed for MI classification in BMI. Imagery signal classification is performed by LR method. KNN is utilized in seizure detection, where NB is utilized for detecting the lower limb movement by analyzing EEG signals [8]. At the same time, DT is primarily utilized for hand amplitude modulation and movement interpretation spatial activity. Deep Learning (DL) method could considerably simplify processing channel, allow automated end-to-end training of retrieval, preprocessing, and classification models [9], while guaranteeing better performance in target. Deep neural network (DNN) stimulated by previous methods like multilayer perceptron (MLP).

This study designs an arithmetic optimization with RetinaNet based deep learning model for MI classification (AORNDL-MIC) technique on BCIs. The proposed AORNDL-MIC technique undergoes two stages of reprocessing namely Multiscale Principal Component Analysis (MSPCA) based denoising and Continuous Wavelet Transform (CWT) based decomposition. Besides, the arithmetic optimization algorithm (AOA) based RetinaNet model is as feature extractor which are then classified by the use of ID3 classifier. To ensure the better results of the AORNDL-MIC approach, a number of experiments were carried out and the result is inspected under different aspects.

The rest of the paper is organized as follows.  Section 2 offers related works, Section 3 provides proposed model, Section 4 discusses performance validation, and Section 5 draws conclusion.

## 2. Related Works

Zhang et al. [10] validate and developed a DL-based algorithm for automatically recognizing two distinct MI states by choosing the related EEG channel. It employs an automated channel selection (ACS) approach. Furthermore, we proposed a CNN method for fully exploiting the time-frequency feature, therefore outperforming conventional classification method interms of robustness and accuracy. Kant et al. [11] present an integration of DL-based TL and CWT for solving the problems. CWT transforms 1D-EEG signal into 2D time-frequency-amplitude representation enables users to make use of deep network via TL method. Corsi et al. [12] adapted a fusion technique that integrates features from instantaneously recorded MEG and EEG signals to enhance classification performance in MI-based BCI. Thomas et al. [13] introduce a discriminatory filter bank (FB) common spatial pattern model for extracting FB for the classification of MI. The presented model improves the classifier performance in BCI datasets.

Dong et al. [14], proposed a hierarchical SVM approach for addressing an EEG-based 4-class MI classification process. Wavelet packet transform is applied for decomposing original EEG signal. EEG feature vector is extracted and a a two-layer HSVM approach is developed for classifying this EEG feature vector, whereas “OVO” classifier is utilized in the initial layer as well as “OVR” in the next layer. Zhang et al. [15], proposed a “brain-ID” architecture based hybrid DNN using TL method for handling single difference of 4-class MI tasks. A dedicated HDNN is designed for learning the common feature of MI signals. The suggested algorithm comprises LSTM and CNN models that are employed for decoding the spatiotemporal features of the MI signal. Zhang et al. [16] introduce 5 systems for adoptation of a DCNN based EEG-BCI scheme for decoding hand MI. All the systems are widely trained, pretrained method and adapt it to improve the efficiency.

## 3. The Proposed Model

In our study, an AORNDL-MIC approach was introduced to classify the MI on BCIs. The proposed AORNDL-MIC technique encompasses a series of operations namely MSPCA based denoising, CWT based decomposition, RetinaNet based feature extraction, AOA based hyperparameter tuning, as well as ID3 based classification.

### 3.1. Data Preprocessing

Initially, the data preprocessing takes place in two stages namely MSPCA based noise removal and CWT based decomposition. Consider a measurement data set with *m* sensor exists, namely *xeR*^*m*^. All the sensors in the measurement samples have *n* sampling data, that is integrated into a data matrix of size *mxn*. The procedure has been shown as follows [2]:

(1) $$\begin{array}{c} X=\left[x_{1},x_{2},x_{3},\ldots ,x_{n}\right]. \end{array}$$

All the columns represent a measurement variable, and all the rows of *X* denote a sample. The PCA models initiated by normalizing all the samples of *X* by calculating the covariance matrix of *X*.

(2) $$\begin{array}{c} cov\left(x\right)≂\frac{X^{T}.X}{n-1}. \end{array}$$

The method of decomposition *X* in its PCA, in which *PeR*^*m*×*A*^ has initial *A* feature vector of cov (x). Once the feature decomposition of *X* is made, the size of feature value is arranged from larger to smaller. *A* indicates the amount of PCA, and it is equivalent to the amount of columns in *T*.*T* ∈ *R*^*m*×*A*^ denotes a matrix, in which all the columns are called as the principal element variable.

(3) $$\begin{array}{c} \left\{\begin{array}{c} X=\hat{X}+Er=T.P^{T}+Er,\\ T=X.P. \end{array}\right) \end{array}$$

In which *λ*_1_, *λ*_2_,…, *λ*_*n*_ represent the initial *A* large eigen values of covariance matrix of *X*, equation (4) is utilized for determining the principal component covariance,

(4) $$\begin{array}{c} \Lambda =\frac{X^{T}.X}{n-1}=\left[\begin{array}{cccc} \lambda_{1} & \ldots & \ldots & \ldots \\ \ldots & \lambda_{2} & \ldots & \ldots \\ \ldots & \ldots & \ldots & \ldots \\ \ldots & \ldots & \ldots & \lambda_{n} \end{array}\right]. \end{array}$$

In the study, the wavelet transform is integrated into the PCA model for creating MSPCA to the incoming signal denoising purpose. In MSPCA, the PCA ability for extracting covariance among parameters is integrated to orthonormal wavelets' capability. The capability of PCA is improved by integrating the multi-scale analysis. Simultaneously, it leads to the MSPCA [17]. It finds linearly correlated wavelet coefficient at multilevel sub-bands, attained using wavelet transform. It represents every subband with less features when eliminating the autocorrelated coefficient. The signal is recreated by utilizing the wavelet syntheses. It reduces unnecessary noises from the received signals and generated noise‐free and simple signal versions. Also, it can be utilized as a scalogram that is signified by exact value of CWT of the signals. MI signal is gradually changing event peppered by abrupt transient with feature taking place at distinct scales, so lower frequency event, offering maximum time localization to higher frequency, shorter duration event, and higher frequency localization to extended duration, is attained utilizing scalogram.

### 3.2. RetinaNet Based Feature Extraction

Next to the data preprocessing phase, the AORNDL-MIC technique involves the RetinaNet model as a feature extractor. RetinaNet comprises of two fully convolution networks (FCN), a feature pyramid network (FPN), and residual network (ResNet). ResNet uses distinct network layers. The important role of ResNet is the concept of RL that enables raw input data to be transferred directly to the succeeding layers. The widely employed type of network layer consists of 101‐layer, 152‐layer, and 50‐layer. The study chooses 101‐layers with the optimal training efficiency [18]. Then, extracted the feature of the echocardiography with ResNet and later transmitted to the following subnetworks. FPN is an approach to effectively extract the feature of all the dimensions in a picture with a traditional CNN.  Figure 1 illustrates the overview of CNN. Firstly, use single‐dimension images as input to ResNet. Next, start from another layer of the convolution network, the feature of each layer was chosen using the FPN and later integrated to generate the last output. The class subnetwork in the FCN implemented the classifier process. Focal loss: it is an amended form of binary cross‐entropy expression, as well as the cross‐entropy loss:

(5) $$\begin{array}{c} CE\left(p,y\right)=\left\{\begin{array}{cc} -\text{log}\left(p\right), & \text{if }y=1,\\ -\text{log}\left(1-p\right), & \text{otherwise,} \end{array}\right) \end{array}$$

whereas *y* ∈ [±, 1] characterizes the ground truth category and *p* ∈ [0,1] signifies the predicted likelihood of algorithm for *y*=1.

(6) $$\begin{array}{c} p_{t}=\left\{\begin{array}{cc} p, & \text{if }y=1,\\ 1-p, & \text{otherwise}. \end{array}\right) \end{array}$$

The abovementioned equation is abbreviated as

(7) $$\begin{array}{c} CE\left(p,y\right)=CE\left(p_{t}\right)=-\log\left(p_{t}\right). \end{array}$$

To resolve the problems of the data imbalance among the negative and positive instances, the novel version is changed into the subsequent form:

(8) $$\begin{array}{c} CE\left(p_{t}\right)=-\alpha_{t}\text{log }\left(p_{t}\right), \end{array}$$

and amongst them,

(9) $$\begin{array}{c} \alpha_{t}=\left\{\begin{array}{cc} \alpha , & \text{if }y=1,\\ l-\alpha , & \text{otherwise,} \end{array}\right) \end{array}$$

whereas, *α* ∈ [0,1] characterizes the weight factor. To resolve the problems of complex samples, the variable *C* is presented for obtaining the last form of focal loss [19].  Figure 2 illustrates the structure of RetinaNet.

(10) $$\begin{array}{c} FL\left(p_{t}\right)=-\alpha_{t}{\left(1-p_{t}\right)}^{\gamma }\text{log }\left(p_{t}\right). \end{array}$$

Since the hyperparameters of the RetinaNet model influence the overall classifier results of the AORNDL-MIC technique, the AOA is utilized. In general, as other MH approaches, the AOA consists of, exploration, and exploitation phases, stimulated by mathematical operations, like −, +, *∗*, and /. Firstly, the AOA generates a set of *N* solutions [20]. Therefore, solution or agent represents *X* population, as:

(11) $$\begin{array}{c} X=\left[x_{N-1,1}x_{N,1}x_{2,1}x_{1,1}x_{N-1,j}x_{N,j}x_{2,j}x_{1,j}x_{N,n-1}x_{1,n-1}x_{N-1,n}x_{N,n}x_{2,n}x_{1,n}\right],\\ X=\left[\begin{array}{ccccc} x_{1,1} & \cdots & x_{1,j} & x_{1,n-1} & x_{1,n}\\ x_{2,1} & \cdots & x_{2,j} & \cdots & x_{2,n}\\ \cdots & \cdots & \cdots & \cdots & \cdots \\ \vdots & \vdots & \vdots & \vdots & \vdots \\ x_{N-1,1} & \cdots & x_{N-1,j} & \cdots & x_{N-1,n}\\ x_{N,1} & \cdots & x_{N,j} & x_{N,n-1} & x_{N,n} \end{array}\right]. \end{array}$$

### 3.3. AOA Based Hyperparameter Tuning

Then, the fitness function of solution is calculated for detecting optimal one *X*_*b*_. According to the Math Optimizer Accelerated (*MOA*) values, AOA implements exploitation or exploration methods. Subsequently, *MOA* is upgraded by

(12) $$\begin{array}{c} MOA\left(t\right)=\text{ Min }+t\times \left(\frac{{\text{Max}}_{MOA}-{\text{Min}}_{MOA}}{M_{t}}\right), \end{array}$$

where *M*_*t*_ characterizes the overall amount of iterations. Min_*MOA*_ and Max_*OA*_ signify the minimal and maximal values of the accelerated function, correspondingly, the division (D) and multiplication (M) are applied in the exploration stage of the AOA, as follows:

(13) $$\begin{array}{c} X_{i,j}\left(t+1\right)=\left\{\begin{array}{c} X_{bj}÷\left(M_{OP}+\in \right)\times \left(\left(UB_{j}-LB_{j}\right)\times \mu +LB_{j}\right),\;r_{2}<0.5,\\ X_{bj}\times M_{OP}\times \left(\left(UB_{j}-LB_{j}\right)\times \mu +LB_{j}\right),\text{ otherwise}. \end{array}\right) \end{array}$$

Next *e* signifies smaller integer value, *LB*_*j*_ and *UB*_*j*_ shows upper and lower limits of the searching space at *jth* parameter. *μ*=0.5 denotes the control function. Furthermore, Math Optimizer (*M*_*OP*_) is determined by

(14) $$\begin{array}{c} M_{OP}\left(t\right)=1-\frac{t^{1/\alpha }}{M_{t}^{1/\alpha }}. \end{array}$$

*α*=5 characterizes the dynamic variable which defines the accuracy of the exploitation stage.

Additionally, subtraction (D) and addition operator (A) operators are employed for executing the AOA exploitation phase, as follows.

(15) $$\begin{array}{c} x_{i,j}\left(t+1\right)=\left\{\begin{array}{c} X_{bj}-M_{OP}\times \left(\left(UB_{j}-LB_{j}\right)\times \mu +LB_{j}\right),\;r_{3}<0.5,\\ X_{bj}+M_{OP}\times \left(\left(UB_{j}-LB_{j}\right)\times \mu +LB_{j}\right),\text{ otherwise}. \end{array}\right) \end{array}$$

Now *r*_3_ characterizes an arbitrary value in [0, 1]. Next, the agent updating procedure is executed by the AOA operator [21]. In summary, Algorithm 1 demonstrates the steps included in AOA.

### 3.4. ID3 Based Classification

Lastly, the ID3 architecture receives the feature vector as input and carries out the classification process. The ID3 technique selects test elements with computing and relating its information gains (IG). Assume *S* be the group of data instances. Supposing the class element *C* has *m* distinct values that signify *m* various class labels *C*_*i*_(*i*=1,2,   …,  *m*). Assume that *S*_*i*_ be the amount of instances from class *C*_*i*_(*i*=1,2,   …,  *m*). The predictable data amount needed for classifying *S* was provided in equation (15):

(16) $$\begin{array}{c} I\left(S_{1},S_{2},\ldots ,S_{m}\right)=-\overset{m}{\underset{i=1}{\sum }}p_{i}{\text{log}}_{2}p_{i}, \end{array}$$

where *p*_*i*_ signifies the probability of samples from *S* appropriate to class *C*_*i*_.*I*(*S*_1_,  *S*_2_,   …,  *S*_*m*_) refers to the average data amount needed for identifying the class label to every instance from S.

Let the element *A* has *v* distinct values {*a*_1_, *a*_2_,…, *a*_*ν*_} from the trained data set S. When *A* is a nominal element, Afterward, the element separates *S* as to *v* subset such that {*S*_1_,  *S*_2_,   …,  *S*_*ν*_}, in that *S*_*j*_ represents the subset of *S* where sample from *S*_*j*_ has the similar element value *a*_*j*_ on *A*. But, instance from *S*_*j*_ can have various class labels [22]. Assume *S*_*ij*_ be the group of instances that class label is *C*_*i*_ from the subset of {*S*_*j*_*|A*=*a*_*j*_, *j* ∈ 1,2,…, *ν*, *S*_*j*_ ∈ *S*} in which element *A*=*a*_*j*_. The needed data amount (i.e., entropy) of element *A* for splitting the trained data set *S* was measured by (16):

(17) $$\begin{array}{c} E\left(A\right)=\overset{\nu }{\underset{j=1}{\sum }}\left(\frac{\left(s_{1j}+s_{2j}+\ldots +s_{mj}\right)}{s}\times I\left(s_{1j},\;s_{2j},\;\ldots ,\;s_{mj}\right)\right). \end{array}$$

The minimum data amount needed, a further purity of sub‐dataset is.

(18) $$\begin{array}{c} I\left(s_{1j},\;s_{2j},\;\ldots ,\;s_{mj}\right)=-\overset{m}{\underset{i=1}{\sum }}p_{ij}{\text{log}}_{2}\left(p_{ij}\right), \end{array}$$

where *p*_*ij*_ implies the probability of instances from *S*_*j*_ based on class *C*_*i*_.*I*(*s*_1*j*_,  *s*_2*j*_,   …,  *s*_*mj*_) signifies the average data amount needed for identifying the class labels to every instance from *S*_*j*_. The IG of *A* has determined as:

(19) $$\begin{array}{c} \text{Info Gain }\left(A\right)=I\left(S_{1},\;S_{2},\;\ldots ,\;S_{m}\right)-E\left(A\right). \end{array}$$

Specifically, the count of novel data requirement (only dependent upon class) minus the count of novel data requirements (based the split on element *A*). Selecting the element with maximal Info Gain (A) as test element that is allocated to internal node from DT. During this process, the required data amount to classify samples is minimal.

## 4. Results and Discussion

The performance validation of the AORNDL-MIC technique has been validated under two dataset includes BCI competition 2003 dataset III and BCI competition IV data set 2b. The BCI competition 2003, dataset III [23], comprises 3-channel EEG data in healthy females, for the imagination of the right, and left -hand movements. The data from the analysis has of recording in the motor cortex area of brain utilizing 3 electrodes (C3, Cz, and C4) under the motor imagery of combined right-or-left-hand movement. All individual trail last to 9-second duration of data to all channels C3, Cz, and C4 per trial with every label obtainable. It holds 280 out of which 140 trials were accessible with its labels, and other 140 instances were employed for validation method. The BCI competition IV data set 2b comprises nine subjects all with 5 sessions of motor imagery experimentally, amongst that the initial 2 sessions are verified with no feedback and the remaining 3 sessions are combined online feedback [24].

### 4.1. Result Analysis on BCI Competition 2003 III Dataset

Figure 3 illustrates the confusion matrices generated by the AORNDL-MIC algorithm under five iterations. At iteration-1, the AORNDL-MIC technique has identified 67 instances in left class and 68 instances in right class. Moreover, at iteration-3, the AORNDL-MIC method has identified 69 instances into left class and 68 instances into right class.

Furthermore, at iteration-5, the AORNDL-MIC approach has identified 67 samples into left class and 66 samples into right class.

Table 1 and Figures 4, 5 provides a classifier results of the AORNDL-MIC algorithm on BCI competition 2003 III dataset. The experimental result indicates the better outcomes of the AORNDL-MIC technique under each iteration. For example, with iteration-1, the AORNDL-MIC algorithm has gained precision of 97.10%, recall of 95.71%, accuracy of 94.43%, *F* − score of 96.40%, and kappa of 95.26%. Meanwhile, with iteration-3, the AORNDL-MIC method has reached precision of 97.18%, recall of 98.57%, accuracy of 97.86%, *F* − score of 97.87%, and kappa of 97.13%. Eventually, with iteration-5, the AORNDL-MIC system has obtained precision of 94.37%, recall of 95.71%, accuracy of 95%, *F* − score of 95.04%, and kappa of 93.30%.

A comparative analysis of the AORNDL-MIC approach with current methodologies on the test BCI competition 2003, dataset III showed in Figure 6 and Table 2. The result exhibits that the SqueezeNet, ResNet50, GoogleNet, DenseNet201, ResNet18, and ResNet101 techniques have resulted to lower kappa values of 57%, 41%, 44%, 36%, 29%, and 30% correspondingly. Next, the VGG19, AlexNet, and VGG16 models have resulted in slightly increased kappa values of 91%, 87%, and 90%, respectively. However, the proposed AORNDL-MIC technique has accomplished higher kappa value of 94.84%.

A comparative study of the AORNDL-MIC method with recent algorithms on the test BCI competition 2003, dataset III is illustrated in Table 3 and Figure 7. The outcome demonstrates that the CSP-SVM, STFT-KNN, Optimized GA FKNN-LDA, Hybrid KNN, and WTSE-SVM techniques have resulted in minimum accuracy values of 82.86%, 83.57%, 84%, 84.29%, and 86.40%, respectively. Then, the Adaptive PP-Bayesian, STFT-DL, and CWTFB-TL methods have resulted in slightly maximal accuracy values of 90%, 90%, and 95.71% correspondingly. Lastly, the proposed AORNDL-MIC method has accomplished superior accuracy value of 96.14%.

### 4.2. Result Analysis on BCI Competition IV Data Set 2b Dataset

A classification results of the AORNDL-MIC method on BCI competition IV data set 2b under several subjects and runs is shown in Table 4 and Figure 8. The experimental value indicates that the AORNDL-MIC algorithm has demonstrated better performance with an average accuracy of 85.33%, 84.22%, 90.11%, 87.11%, and 85.89% under runs 1–5, respectively.

An average classification results of the AORNDL-MIC method under several subjects are portrayed in Figure 9. The results showed that the AORNDL-MIC system has the ability of accomplishing improved outcomes with the maximum average accuracy of 81.20% under S-1, 87.20% under S-2, 84.60% under S3, 91.60% under S-4, and so on.

Table 5 and Figure 10 provide a comparative study of the AORNDL-MIC system with current methodologies interms of accuracy. The experimental results indicated that the AORNDL-MIC technique has resulted in better results over the other methodologies under all subjects. For instance, with S-1, the AORNDL-MIC algorithm has accomplished higher performance of 81.20% whereas the CSP, FBCSP MIBIF, FBCSP MIRSR, and FDBN techniques have attained lower accuracy of 66%, 68%, 70%, and 81% respectively. Moreover, with S-5, the AORNDL-MIC approach has reached superior accuracy of 85.80% whereas the CSP, FBCSP MIBIF, FBCSP MIRSR, and FDBN methods have attained lesser accuracy of 77%, 93%, 93%, and 93%, respectively. Furthermore, with S-9, the AORNDL-MIC approach has gained superior accuracy of 87.60% whereas the CSP, FBCSP MIBIF, FBCSP MIRSR, and FDBN methods have achieved minimum accuracy of 83%, 88%, 87%, and 91% correspondingly.

For ensuring the improvement of AORNDL-MIC model, an average accuracy analysis is also made in Figure 11. From the figure, it is apparent that the CSP and FBCSP MIBIF techniques have reached lower performance with an average accuracy of 76.33% and 79.56% respectively. In line with, the FBCSP MIRSR and FDBN systems have resulted in moderately increased average accuracy of 80.22% and 84.22% respectively. However, the AORNDL-MIC approach has gained effective performance over the other methodologies with the maximal average accuracy of 86.53%. By observing the experimental results and discussion, it is confirmed that the AORNDL-MIC approach has shown better results over the other methodologies.

## 5. Conclusion

In this study, an AORNDL-MIC system was developed to categorize MI on BCIs. The proposed AORNDL-MIC technique encompasses a series of operations namely MSPCA based denoising, CWT based decomposition, RetinaNet based feature extraction, AOA based hyperparameter, and ID3 based classification. The AOA is employed to tune the hyperparameter of RetinaNet and improves the classification performance of the AORNDL-MIC technique. For ensuring the outcome of the AORNDL-MIC method, a number of experiments were performed and the outcome is examined under different aspects. The experiment results of the AORNDL-MIC algorithm on the benchmark datasets reported its promising outcome over the current state of art approaches. In the future, hybrid DL model can be utilized for boosting the efficacy of the MI classification process.

## Figures and Tables

**Figure 1:** Overview of CNN.

**Figure 2:** RetinaNet network architecture.

**Figure 3:** Confusion matrix of AORNDL-MIC technique under five iterations.

**Figure 4:** Result analysis AORNDL-MIC technique on BCI competition 2003 III datasets.

**Figure 5:** Average analysis AORNDL-MIC technique on BCI competition 2003 III dataset.

**Figure 6:** Kappa analysis of AORNDL-MIC technique with current approaches.

**Figure 7:** Accuracy analysis of AORNDL-MIC approach with current methodologies.

**Figure 8:** Training accuracy analysis of AORNDL-MIC technique.

**Figure 9:** Average training accuracy analysis of AORNDL-MIC technique.

**Figure 10:** Accuracy analysis of AORNDL-MIC technique with recent methods.

**Figure 11:** Average Accuracy analysis of AORNDL-MIC algorithm with current methodologies.

**Algorithm 1:** Pseudocode of AOA.

**Table 1:** Classification outcomes of AORNDL-MIC approach on BCI competition 2003 III datasets.

No. of iterations	Precision	Recall	Accuracy	F-score	Kappa
Iteration-1	97.10	95.71	96.43	96.40	95.26
Iteration-2	97.10	95.71	96.43	96.40	95.26
Iteration-3	97.18	98.57	97.86	97.87	97.13
Iteration-4	93.15	97.14	95.00	95.10	93.24
Iteration-5	94.37	95.71	95.00	95.04	93.30
Average	95.78	96.57	96.14	96.16	94.84

**Table 2:** Kappa analysis of AORNDL-MIC technique with existing approaches on test BCI competition 2003, dataset III.

Methods	Kappa
AORNDL-MIC	94.84
VGG19	91.00
AlexNet	87.00
VGG16	90.00
SqueezeNet	57.00
ResNet50	41.00
GoogleNet	44.00
DenseNet201	36.00
ResNet18	29.00
ResNet101	30.00

**Table 3:** Accuracy analysis of AORNDL-MIC technique with existing approaches on test BCI competition 2003, dataset III.

Methods	Accuracy
Hybrid KNN	84.29
CSP-SVM	82.86
Adaptive PP-Bayesian	90.00
STFT-KNN	83.57
STFT-DL	90.00
Optimized GA FKNN-LDA	84.00
WTSE-SVM	86.40
CWTFB-TL	95.71
AORNDL-MIC	96.14

**Table 4:** Classification results of the AORNDL-MIC approach under several subjects and runs.

No. of runs	S-1	S-2	S-3	S-4	S-5	S-6	S-7	S-8	S-9	Avg.
R-1	87.00	85.00	88.00	86.00	84.00	76.00	83.00	96.00	83.00	85.33
R-2	71.00	83.00	80.00	94.00	85.00	79.00	91.00	83.00	92.00	84.22
R-3	84.00	96.00	94.00	98.00	88.00	90.00	85.00	89.00	87.00	90.11
R-4	82.00	91.00	75.00	89.00	91.00	92.00	81.00	88.00	95.00	87.11
R-5	82.00	81.00	86.00	91.00	81.00	87.00	95.00	89.00	81.00	85.89
Avg.	81.20	87.20	84.60	91.60	85.80	84.80	87.00	89.00	87.60	86.53

**Table 5:** Comparative study of AORNDL-MIC technique with recent methodologies interms of accuracy.

Subject	CSP	FBCSP MIBIF	FBCSP MIRSR	FDBN	AORNDL-MIC
S-1	66.00	68.00	70.00	81.00	81.20
S-2	62.00	59.00	61.00	65.00	87.20
S-3	57.00	59.00	61.00	66.00	84.60
S-4	97.00	98.00	98.00	98.00	91.60
S-5	77.00	93.00	93.00	93.00	85.80
S-6	75.00	80.00	81.00	88.00	84.80
S-7	77.00	78.00	78.00	82.00	87.00
S-8	93.00	93.00	93.00	94.00	89.00
S-9	83.00	88.00	87.00	91.00	87.60
Average	76.33	79.56	80.22	84.22	86.53

## Data Availability

Data sharing not applicable to this article as no datasets were generated during the current study.
